RETRACTED

# A Meta-Analysis of CT as a Tool for Diagnosing and Treating Shoulder Joint Bankart Injuries

**DOI:** 10.1155/2022/9137706

**Published:** 2022-08-18

**Authors:** Yibin Yang, Longqiang Zou, Zhengnan Li

**Affiliations:** Department of Sports Medical, Ganzhou People's Hospital & the Affiliated Ganzhou Hospital of Nanchang University, Ganzhou, 341000 Jiangxi Province, China

## Abstract

**Objective:**

The shoulder joint is the most flexible joint in the human body. It is a typical multiaxial ball-and-socket joint. The humeral head is approximately spherical, and the glenoid is small and shallow. This article mainly discusses the application value of computerized tomography (CT) in the early diagnosis of skeletal Bankart injury of the shoulder joint.

**Methods:**

The chemical quality was evaluated according to the physical therapy evidence database PEDro scale. The literature quality evaluation scale and the NO scale are also used to evaluate the quality of each nonrandomized study. The standard quality scores of the literature quality evaluation scale are as follows: (1) the selection of the study group; (2) the comparability of the study group; and (3) (cohort study) clear interest results. Outcome measurement: Postoperative shoulder joint stability and range of motion (ROM) are the main results of Bankart injury patients undergoing open repair surgery and arthroscopic repair surgery. The secondary results of the survey included the Rowe score, the shoulder stability score, the American shoulder and elbow surgery score ASES, the University of California, Los Angeles, shoulder score UCLA, and the operation time.

**Results:**

Four of the included studies are randomized controlled trials, and the other studies are cohort studies. After meta-analysis, a fixed-effect model (*I*^2^ = 34%) was used to observe the difference in shoulder stability treatment between the two groups and was statistically significant (*P* = 0.008, RR = 0.94, 95% confidence interval: 0.89~0.98). The analysis results showed that compared with patients undergoing open surgery, patients' undergoing arthroscopic repair had better postoperative shoulder motion range (*P* < 0.001, SMD = 0.47, 95% confidence interval: -0.72~0.22), and there is no significant heterogeneity.

**Conclusion:**

The Bankart injury of the shoulder joint cannot be diagnosed by X-ray examination alone due to its anatomical location and the size of the fracture fragments. CT examination has a better auxiliary diagnostic effect in the early stage of skeletal Bankart injury.

## 1. Introduction

The shoulder joint is a typical multiaxis ball and socket joint. The glenoid labrum made of fibrocartilage around the glenoid deepens the depth of the joint socket, but still only accommodates 1/4-1/3of the humeral head. This structure of the shoulder joint determines a greater range of joint motion, but also reduces the stability of the joint. When the shoulder joint is dislocated, the humeral head is often removed from the lower part. Sliding out, dislocation of the front lower part occurred. The incidence of shoulder dislocation injury is relatively high for people who have been doing heavy physical activity and physical exercise for a long time. Shoulder dislocation brings great pain and inconvenience to patients' life and work. The incidence of skeletal Bankart injury in patients with recurrent shoulder dislocation can reach 41%. Bone Bankart injury is caused by traumatic avulsion of the anterior inferior labrum of the shoulder joint or recurrent unstable shoulder dislocation accompanied by a large bony labrum defect. It is common in anterior shoulder dislocation caused by traumatic factors or anterior inferior dislocation, and the incidence of this injury in clinical work is relatively high, accounting for 5.4%-70% of shoulder instability caused by traumatic factors [1–5]. Due to traumatic factors, the anterior and inferior glenoid bone defects are caused. The glenoid loses its normal structural characteristics and becomes an “inverted pear-shaped” structure. The humeral head and glenoid lose their normal contact relationship during activities, and joints such as shoulder dislocation occur. Unstable performance. Bankart injury first appeared in 1938 in a report of 27 patients with anterior shoulder instability due to Bankart injury. This injury was caused by the avulsion of the anterior and lower labrum of the shoulder joint, and the general impact did not exceed the 35-year-old crowd. Traditional open Bankart repair surgery is recognized by many surgeons as a recognized standard treatment [6].The traditional open Bankart repair surgery has been proven to significantly improve the stability of the shoulder joint. After this type of surgery, the recurrence rate of patients is less than 10% [7], and the low failure rate of the operation reaches 0-11% [8]. However, limited external rotational activity and secondary osteoarthritis are disadvantages of open surgery. The description of Bankart repair surgery under arthroscopic surgery appeared for the first time in 1993 [9]. In the past two decades, with the development of science and technology, related instruments and surgical implants suitable for arthroscopic surgery have been continuously updated, and with the improvement of surgeons' experience in arthroscopic surgery, arthroscopic Bankart repair surgery has gradually been advocated by some surgeons [10]. Compared with open surgery, arthroscopic surgical treatment has some advantages, such as smaller skin incisions, short operation time, reduced postoperative pain, and reduced complication rate [11]. However, some survey reports show that arthroscopic surgery has a relatively higher recurrence rate compared with standard open surgery [12]. In addition, arthroscopic techniques require experienced surgeons with relatively long learning periods and expensive instruments. So far, some of the newer techniques of arthroscopic repair surgery, such as suture anchor fixation, have the same failure rate as the traditional standard open surgery. However, these available data come from short-term and mid-term follow-up, not long-term follow-up data. Therefore, there is a lack of strong evidence-based medical evidence to determine which surgical method has better clinical effects for patients with skeletal Bankart injury of the shoulder. Some authors have concluded that open repair surgery has a lower recurrence rate, but others believe that there is no significant difference in failure rate between standard open surgery and arthroscopic Bankart repair surgery. In addition, some new high-quality studies have recently been published [13].Therefore, we conducted this meta-analysis to determine which surgical method has a better clinical effect for Bankart injury treatment. In conclusion, Bankart injury cannot be diagnosed by X-ray alone because of its anatomic location and fracture fragment size. CT examination has a better auxiliary diagnostic effect in the early stage of skeletal Bankart injury.

RETRACTED

## 2. Materials and Methods

### 2.1. Search Strategy

The correlation in CT as a tool for diagnosing and treating shoulder joint Bankart injuries was searched through the online databases Pub Med (1966 to December 2016) and EMBASE (1966 to December 2016). Only published studies in English are included. The articles in the reference catalogue that may meet the conditions are also checked. The keywords used to search for are as follows: anterior instability of the shoulder joint, Bankart injury, dislocation, and subluxation. To avoid duplication, if multiple research articles include the same number of patients, the results are summarized.

### 2.2. Inclusion Criteria

In the literature, DSA and surgery are the gold standards, and double-blind evaluation is used. The patients included in the study are comprehensive, and the included literature has the original number data, can directly or indirectly obtain true and false positive numbers, true and false negative numbers or sensitive data such as degree, specificity, etc. have not been published repeatedly, and the sample size is larger than 10.

RETRACTED

### 2.3. Evaluation of the Literature Quality of the Included Studies

According to QUADAS2 (Review Manager5.2), independent literature quality evaluation was made for each included literature. When there is a disagreement, negotiate or refer to a third party to resolve.

### 2.4. Data Extraction

Two authors independently checked the titles and titles of the retrieved documents according to the inclusion criteria. A preliminary screening of the abstract is carried out. After the preliminary screening, read the full text carefully to eliminate poor quality. For incomplete data and repetitive articles, if there are disagreements, we will agree to quotient solution. Extracted data includes the researcher, the publication year of the paper research, the country where the person is located, the inspection equipment, the number of patients, the reference standard, the inspection department Bits, the number of true and false positives, and the number of true and false negatives.

### 2.5. Statistical Processing

Meta-disc 1.4 software was used for statistical analysis. The heterogeneity test level is *a* = 0.1; combined with the magnitude of Iz heterogeneity, Iz G25% is less heterogeneity; 250oGIzG50% is moderate heterogeneity; Iz-50% represents high heterogeneity of research findings. If there is no heterogeneity, combine the effect size, and use Meta-discl. 4 to draw the summary receiver operating characteristic curve (SROC). If the heterogeneity of the included studies is obvious, analyze the reasons for the heterogeneity, and only conduct a descriptive analysis.

### 2.6. Inspection Method

Radiology and CT were used to quantify bone loss. Radiographic examination can be used to examine patients with severe pelvic bone loss. CT imaging has good evidence for accurate quantification of pelvic bone loss, shoulder X-ray, and chest fluoroscopy; CT examination of the shoulder joint: The patient lies on his back, with the affected limb straightened down, and scans from the upper edge of the clavicle to 1/2 of the humerus, with a layer thickness of 3 mm. The results of the imaging examination were read independently by an imaging physician and an orthopedic physician.

#### 2.6.1. Result Measurement

The stability and range of motion (ROM) of the shoulder joint after surgery are the main results of Bankart injury patients undergoing open repair surgery and arthroscopic repair surgery. If the patient does not observe dislocation or subluxation of the shoulder joint after surgery, or the fear test is negative, then the shoulder joint is considered stable. The range of motion ROM mainly includes the loss of the range of the external rotation angle when the arm is extended at 90°. The secondary results of the survey included the Rowe score [14], the shoulder stability score [15], the American shoulder and elbow surgery score ASES [16], the University of California, Los Angeles, shoulder score UCLA [17], and the operation time.

RETRACTED

#### 2.6.2. Inclusion Criteria

1. Published English literature
2. Comparison of open repair surgery and arthroscopic repair surgery for shoulder joint stability in Bankart injured patients

Qualitative

(3) All patients are 18 years old or above
(4) Follow-up for at least 2 years
(5) There are available shoulder joint injury and dislocation recurrence data and shoulder function score

#### 2.6.3. Exclusion Criteria

1. Nonpublished English documents
2. The study was followed up for less than 2 years
3. Insufficient original data for meta-analysis
4. In vitro studies or noncontrast studies
5. Research objects include patients younger than 18 years old
6. The sample size is less than 50

#### 2.6.4. Research Methods

Search the online databases Pub Med (1966 to December 2019) and EMBASE (1966 to December 2019). Only published studies in English are included. The articles in the reference catalogue that may meet the conditions are also checked. The keywords used to search for are as follows: anterior instability of the shoulder joint, Bankart injury, dislocation, and subluxation. To avoid duplication, if multiple research articles include the same number of patients, the results are summarized. Data extraction and methodological quality evaluation. Data extraction and independent evaluation were carried out by two researchers and verified by a third, more senior researcher. The extracted information includes: (1) the characteristics of the included study, including the author, type of study design, and publication date; (2) including the demographic characteristics of the included subjects, including sample size, age, gender, and duration of follow-up (from injury to surgery time) and details of surgery; and (3) details of the research results. Resolve differences between different authors through discussion. In order to avoid the occurrence of missing necessary data, the authors who are eligible for inclusion in the trial are contacted to obtain relevant data. The methodological quality of each randomized controlled trial (RCT) is evaluated according to the physical therapy evidence database PEDro scale [16]. The literature quality evaluation scale and the NO scale [17] are also used to evaluate the quality of each nonrandomized study. The standard quality scores of the literature quality evaluation scale are as follows: (1) the selection of the study group; (2) the comparability of the study group; and the (3) (cohort study) clear interest results. After a full review, a total of 11 independent studies were included in this meta-analysis, and the cumulative sample size as of the last follow-up was 1, 022. The difference between the two groups was not statistically significant (*P* = 0.08, SMD = –2.01, 95% confidence interval: -4.29 to 0.27), with very significant heterogeneity (*I*^2^ = 97%). Potential publication bias due to study size (tendency for the smaller studies to show larger effects) was explored by plotting the natural logarithm of the estimate of RR (ln RR) versus the inverse of standard error (1/SE). Funnel plot asymmetry was tested using the linear regression method (Figure 1).

RETRACTED

After a full review, a total of 11 independent studies were included in this meta-analysis, and the cumulative sample size as of the last follow-up was 1022. Four of the included studies are randomized controlled trials [18], and the other studies are cohort studies [19].

## 3. Result

All 11 studies evaluated postoperative shoulder stability, including 512 cases in the arthroscopy group and 510 cases in the open group. After meta-analysis, a fixed-effect model (*I*^2^ = 34%) was used to observe the difference in shoulder stability treatment between the two groups was statistically significant (*P* = 0.008, RR = 0.94, 95% confidence interval: 0.89~0.98). Four studies provided ROM data on the range of motion of the shoulder joint.

As a main result of the study, the analysis results showed that patients undergoing arthroscopic repair had better postoperative shoulder motion range, compared with patients undergoing open surgery (*P* < 0.001, SMD = 0.47, 95% confidence interval: -0.72~0.22), with no significant heterogeneity. Meta-analysis showed that there was no significant difference in postoperative functional results for patients with Bankart injury under the two different treatment strategies, and the results were not statistically significant. Rowe score (*P* = 0.16), ASES score (*P* = 0.24), shoulder stability score (*P* = 0.32), and ULCA score (*P* = 0.18).

Data on the number of intraoperative operations were only obtained in 2 trials, including 115 cases in the arthroscopy group and 108 cases in the open group. The difference between the two groups was not statistically significant (*P* = 0.08, SMD = –2.01, 95% confidence interval: -4.29 to 0.27), with very significant heterogeneity (*I*^2^ = 97%). However, patients in the arthroscopic repair group have tendency to reduce the operation time and frequency, compared with patients in the open repair surgery group.

## 4. Discussion

Skeletal Bankart injury of the shoulder joint is a defect caused by traumatic factors such as bone avulsion in the front of the scapular glenoid of the shoulder joint [20, 21]. This result is caused by repeated dislocations of the shoulder joint and continuous wear and tear of the scapular glenoid edge. Recent studies have shown that in recurrent shoulder joint instability caused by trauma, the incidence of skeletal Bankart injury is as high as 90%. Under the action of a small external force, it is enough to make the humeral head prolapse from the glenoid and form a shoulder dislocation. Yang Guohui et al. [22] followed up 88 patients with scapular glenoid Bankart injuries that were clearly diagnosed by imaging. The results of the follow-up study showed that the incidence of poor fracture healing after arthroscopic Bankart repair surgery was 16.6%. The incidence of poor fracture healing was significantly higher in the chronic case group. According to related published literature, there are two main focuses on the repair of bone defects of the shoulder joint skeletal Bankart injury: ①Reduction and fixation of the scapular glenoid avulsion fracture: the fracture often shifts to the inside of the original physiological position to the shoulder and neck. Therefore, it is necessary to restore the displaced scapular glenoid fracture block to the original physiological position at the level of the scapular glenoid articular surface and fix it firmly during the operation. ②When reducing and fixing the anterior scapular glenoid avulsion fracture, tightening the joint capsule tissue in front of the shoulder joint cannot be ignored either. Xiao Lihua et al. [23] classified the skeletal Bankart injury of the shoulder joint based on the imaging data of the patient: type I: the fracture piece is separated from the glenoid, and the joint capsule of the shoulder joint is continuous; type II: the severely displaced bone block is deformed. It is connected to the nonanatomical position of the shoulder glenoid margin; type III is divided into two subtypes, namely, type IIIA anterior labrum bony defect area < 25% and type IIIB anterior labrum bony defect area > 25%.

RETRACTED

Related literature reports that patients with types I and II shoulder joint skeletal Bankart injuries should actively adopt arthroscopic surgery. Type IIIB skeletal Bankart injury with a large and serious bone defect on the scapular glenoid side is mainly used for arthroscopic repair with wire anchors or open surgery with autogenous or allogeneic free bone grafting or Brinstow-Latarjet surgery to reconstruct the physiological bone retaining structure of the scapular glenoid bone defect and maintain the stability of the shoulder joint [24].

With the development of arthroscopic technology and related equipment, there are different ways of fixing free bones of the skeletal Bankart injury of the shoulder joint under arthroscopy with hollow nails and wire anchors. For imaging diagnosis of patients with small scapular glenoid bone injuries, it is advisable to use single-row single-line anchors for displacement and fixation. For imaging diagnosis, it is recommended to use a single row of single-line anchors for displacement and fixation; imaging diagnosis shows that the scapular glenoid defect area is larger for bone injury, in order to achieve shoulder joint anatomy. For reduction and firm fixation, most research results show that the use of double-row double-line anchor fixation surgery is recommended. It is reported in the literature that some scholars have experimental studies on the clinical efficacy comparison of arthroscopic single-row single-line anchors and double-row double-line anchors for repairing skeletal Bankart injury of the shoulder joint [25]. In the study, 14 cases of skeletal Bankart injury models of the shoulder joint were made. There is difference in shoulder stability treatment between the arthroscopy group, and open group was statistically significant, mainly because the treatment method had effect on the shoulder stability.

The area of the scapular glenoid bone defect reached 25%. The study models were divided into 2 groups. One group was repaired with arthroscopic single-row single-line anchors, and the other group was repaired with arthroscopic double anchors. A row of double-line anchor nails is repaired. After the operation, the shoulder joints of the two groups of subjects were subjected to biomechanical tests such as joint movement. The results of the study show that the arthroscopic double-row double-line anchor repair has a better shoulder joint reduction effect than the single-row single-line anchor repair and the zero position of the shoulder joint glenoid is more stable. Kim et al. [26] and Bhatia et al. [27] believe that if the area of the scapular glenoid defect is less than 15%, only the soft tissue of the labrum joint capsule can be repaired to restore the stability of the shoulder joint. Jiang et al. [28] studied whether the anatomical reduction of the shoulder joint skeletal Bankart injury and the repair of displaced fractures and the healing of the bone defect are necessary under arthroscope. The study selected 50 cases of shoulder joint skeletal Bankart injury and recurrent shoulder with a clear diagnosis of imaging. Patients with anterior joint dislocation of the shoulder joint should be treated with arthroscopic reduction and internal fixation with wire anchors. Before and after the operation, the joint range of motion and Constant-Murley and Rowe scores were used to evaluate the shoulder joint function of the patients before and after the operation. The results of the study showed that the postoperative imaging data of 3 of the 4 failed patients showed that the repaired area of the glenoid defect was less than 80%. The repaired area of the glenoid defect was greater than 80% in the successful cases. Some researchers at home and abroad have used Latarjet 2 open surgical methods to treat patients with shoulder glenoid defect area > 25% skeletal Bankart injury or engaging Hill-Sachs injury (coracoid parallel transposition and coracoid process, internal rotation 90°index) [29]. After the operation, ASES score, Constant-Murley score, and visual analog scale (VAS) instability score were used to systematically evaluate the patient's shoulder joint function.

RETRACTED

The results of the study showed that with the open Latarjet surgical treatment plan, the skeletal Bankart-injured shoulder joint can obtain better static stability and effectively reduce the recurrence rate of shoulder dislocation, Comparison of coracoid transposition and coracoid internal surgery. Compared with the 90° rotation and transposition operation, the imaging data of the postoperative follow-up suggest that the fracture healing rate is relatively higher. At present, the best imaging diagnosis method for skeletal Bankart injury of the shoulder joint is MRI, because MRI has the highest sensitivity and accuracy in diagnosing this injury [30]. However, MRI examinations are expensive, and many primary hospitals are not equipped with MRI equipment. In the early stage of injury, MRI has limited soft tissue resolution. Therefore, how to accurately diagnose shoulder skeletal Bankart injuries in limited conditions is an important issue. CT examination can determine whether the patient has a skeletal Bankart injury of the shoulder joint in a short time. When performing CT examinations on such patients, the accuracy of the examination is determined by the thickness of the slice.

In general, 16-slice or 8-slice CT in county-level hospitals can quickly scan and diagnose fractures, and there will be no low-slice CT, a problem with damage diagnosis. It is worth noting that before the application of CT examination, a strict physical examination of the patient is required. If a patient with skeletal Bankart injury of the shoulder is accompanied by fractures of the acromion and coracoid process, the body surface needs to be projected at the corresponding position under the tenderness and on the CT film. Focus on this position to avoid misdiagnosis or missed diagnosis of the disease. In this study, X-ray and CT examinations were performed on 30 cases of shoulder joint skeletal Bankart injuries diagnosed and treated [31]. The results showed that 18 cases were clearly diagnosed by X-ray, with a diagnosis rate of 60.00%; CT diagnosis accuracy rate was 96.67%, and CT observations found that 30 patients had fractures of different degrees in the front of the glenoid, accompanied by different degrees of displacement. CT examinations can be seen that the information provided is more detailed and the results are more accurate. In addition, MRI is the only effective inspection method for fibrous Bankart injury. If the patient has been excluded from the bone injury by CT, the shoulder joint activities should be followed up during the immobilization treatment. If there is repeated dislocation of the shoulder joint, MRI should be implemented as soon as possible. Review to fully grasp the condition.

RETRACTED

### 4.1. Research on the Skeletal Bankart Injury of the Shoulder Joint

The shoulder joint is a typical multiaxis ball and socket joint. The head of the humerus is approximately spherical, and the glenoid is small and shallow. The glenoid labrum made of fibrocartilage around the glenoid deepens the depth of the joint socket, but still only accommodates 1/4-1/3 of the humeral head. This structure of the shoulder joint determines a greater range of joint motion, but also reduces the stability of the joint. At the same time, the shoulder joint capsule is thin and loose, and the lower wall is relatively weakest. When the shoulder joint is dislocated, the humeral head is often removed from the lower part. Sliding out, dislocation of the front lower part occurred. The incidence of shoulder dislocation injury is relatively high for people who have been doing heavy physical activity and physical exercise for a long time. Shoulder dislocation brings great pain and inconvenience to patients' life and work. The incidence of skeletal Bankart injury in patients with recurrent shoulder dislocation can reach 41%. Because this type of injury can seriously affect the stability of the shoulder joint and cause repeated dislocations of the shoulder joint, active surgical treatment is required. Bone Bankart injury is caused by traumatic avulsion of the anterior inferior labrum of the shoulder joint or recurrent unstable shoulder dislocation accompanied by a large bony labrum defect. It is common in the anterior dislocation of the shoulder joint caused by traumatic factors or anterior inferior dislocation; the incidence of this injury in clinical work is relatively high, accounting for 5.4%-70% of shoulder instability caused by traumatic factors [32]. Due to traumatic factors, the anterior and inferior glenoid bone defect is caused. The glenoid loses its normal physiological structure and becomes an “inverted pear-shaped” structure. The humeral head and glenoid lose their normal contact relationship during activities, Loss of normal contact between humeral head and pelvis during movement and joint instability in shoulder dislocation. Traditional open Bankart repair surgery is recognized by many surgeons as a recognized standard treatment [33]. The traditional open Bankart repair surgery has been proven to significantly improve the stability of the shoulder joint. After this type of surgery, the recurrence rate of patients is less than 10% [34], and the low failure rate of the operation reaches 0-11%. However, limited external rotational activity and secondary osteoarthritis are disadvantages of open surgery. The description of Bankart's repair surgery under arthroscopy appeared for the first time in 1993. In the past two decades, with the rapid development of arthroscopic instruments and implants and the improvement of surgeons' experience in arthroscopic surgery, arthroscopic surgery Bankart repair surgery is gradually advocated by some surgeons [35]. Compared with open surgery, arthroscopic surgical treatment has some advantages, such as smaller skin incisions, short operation time, reduced postoperative pain, and reduced complication rate. However, some survey reports show that arthroscopic surgery has a relatively higher recurrence rate compared with standard open surgery. In addition, arthroscopic techniques require experienced surgeons with relatively long learning periods and expensive instruments. So far, some of the newer techniques of arthroscopic repair surgery, such as suture anchor fixation, have the same failure rate as the traditional standard open surgery. However, these available data come from short-term and mid-term follow-up, not long-term follow-up data. Therefore, there is a lack of sufficient corroborative medical evidence to determine which surgical method should be used for patients with shoulder joint Bankart injury in order to achieve better clinical results. Although some past studies have summarized the results of published studies comparing standard open surgery and arthroscopic Bankart repair surgery, most of these studies are systematic reviews. Some authors have concluded that open repair surgery has a lower recurrence rate, but others believe that there is no significant difference in failure rate between standard open surgery and arthroscopic Bankart repair surgery. In addition, some new high-quality studies have recently been published.

RETRACTED

### 4.2. The Clinical Research Application Value of Meta-Analysis

Although many medical institutions have begun to use CT to diagnose the early diagnosis of skeletal Bankart injury of the shoulder, a large number of research documents at home and abroad are different due to the uneven geographical, ethnic, and equipment conditions, and the research results are also different. The nine documents included in this study are from different countries. Through screening and quality evaluation of the included documents, the quality level of the included documents is guaranteed, thereby ensuring the reliability of the meta-analysis. In this study, the diagnostic effect indicators of nine documents were combined to increase the statistical power. The combined sensitivity of the included literature was 0.98 (95% CI: 0.96-1.00), indicating that CT can better detect early diagnosis of bone and joint and Bankart injury. The combined specificity is 0.99 (95% CI: (0.97-1.00), indicating that CT diagnoses skeletal Bankart injury of the shoulder. The positive likelihood ratio is the ratio of the true positive rate to the false positive rate, and the negative likelihood ratio is false negative. Therefore, the larger the former, the higher the diagnostic value, and the smaller the latter, the higher the diagnostic value. In this study, the positive likelihood ratio and negative likelihood ratio were 33.14 (95% CI).: 15.74-69.53) and 0.04 (95% CI: 0.02-0.07), both of which indicate that CT has a higher diagnostic value in the early diagnosis of skeletal Bankart injury of the shoulder joint. The diagnostic OR value is that CT has a higher diagnostic value in the early diagnosis of skeletal Bankart injury of the shoulder joint. CT has a higher detection rate of lesions and provides more reliable evidence-based medical evidence. SROC curve is a comprehensive evaluation of the reliability of diagnosis. The SROC curve method performs meta-analysis on multiple diagnostic tests with the same detection target, fits the SROC curve according to the ratio weight, and calculates the area under the SROC curve.

### 4.3. Mate Analysis Heterogeneity Test

By observing the SROC curve plan, it is found that the result does not show a “shoulder-arm”-like distribution, suggesting that there is no threshold effect. In the test of heterogeneity caused by nonthreshold effects, *P* = 0.093 and *I*^2^ = 0%, which proves that there is no heterogeneity caused by nonthreshold effects. In summary, the heterogeneity between the studies is small. Meta-analysis results: Using random effects model, combined effect size, combined sensitivity, specificity, positive likelihood ratio, negative likelihood ratio, and diagnostic OR value were 0.89 (95% CI: 0.96-10.0), 0.99 (95% CI: 0.97-1.00), 33.09 (95% CI: 15.75-69.53), 0.04 (95% CI: 0.02-0.07), and 1110.47 (95% CI: 37.68-3216.73), respectively. There was no statistically significant difference in the combined effect size of each combination. SROC analysis: The area under the SROC curve (AUC) of CT is 0.99, and the Q index is 0.968 (Figure 2).

RETRACTED

Bankart injury of the shoulder joint refers to the avulsion injury of the anterior and inferior shoulder joint glenolabia at the attachment of the anterior inferior glenohumeral ligament complex. It can be accompanied by a fracture of the glenoid edge. After the injury, it is easy to cause instability and habituation in the front of the shoulder joint. Anterior dislocation of the shoulder joint. Burkhart et al. (2000) believe that among patients with a single shoulder dislocation, those without obvious defects in the shoulder glenoid have a 4% risk of redislocation, while those with a glenoid defect are at risk of redislocation. As high as 67%, therefore, the result of skeletal Bankart injury is more serious than that of fibrous Bankart injury. The treatment methods of fibrous Bankart injury and skeletal Bankart injury are also different: Fibrous Bankart injury can be repaired under arthroscopic surgery to obtain good results, and there are also reports on the treatment of fibrous Bankart by incision and repair of the joint capsule labrum. The damage has been well recovered. For patients with skeletal Bankart injury with or without Hill-Sachs injury, arthroscopic repair is more difficult, and for fracture fragments that cannot provide strong fixation, open reconstructive surgery should be considered. The imaging diagnosis of Bankart damage is currently considered to be the most accurate and sensitive MRI examination, and the accuracy and sensitivity of the water-induced three-dimensional VIBE MR reconstruction in the diagnosis of Bankart damage have been greatly improved. However, most primary hospitals are not equipped with MR equipment, and the resolution of early MRI examination of the injury to the soft tissue is limited. How to make an accurate diagnosis of skeletal Bankart injury under limited conditions is very important. Because the consequences of skeletal Bankart injury are more serious, early diagnosis and treatment are more necessary, and the early diagnosis of skeletal Bankart injury has a positive effect on the recovery of surgical treatment. CT examination can determine whether there is bone in a shorter time. The requirements for CT do not need to be as high as those for cardiac CT examinations. The accuracy of the examination mainly depends on the thickness of the layer. Although there is no clear report on the size of the fracture in the front of the glenoid in the Bankart injury, all patients in this group passed CT examination can clarify the location and displacement of fracture injury. Most county-level hospitals can accurately scan the fracture with 8-row and 16-row CT. There is no concern that low-speed CT cannot diagnose skeletal Bankart injuries. However, the CT examination must be established on the premise of a detailed physical examination. Some Bankart injuries are accompanied by fractures such as the coracoid process and acromion. It needs to be established under the tenderness of the body surface projection of the part. Pay attention to its position on the CT film. Effectively avoid the misdiagnosis and missed diagnosis of Bankart injury. For fibrous Bankart injuries, MRI inspection is the only effective inspection method. For patients whose bone injury is excluded by CT, the shoulder joint movement should be observed at the same time of immobilization treatment. If there is repeated shoulder joint dislocation, MRI review and shoulder arthroscopic surgery should be performed. Most patients can get good recovery.

RETRACTED

## 5. Conclusion

The Bankart injury of the shoulder joint cannot be diagnosed by X-ray examination alone due to its anatomical location and the size of the fracture fragments. CT examination has a better auxiliary diagnostic effect in the early stage of skeletal Bankart injury.

## Figures and Tables

**Figure 1:** Funnel plot to evaluate publication bias.

**Figure 2:** The area under the SROC curve.

## Data Availability

The data used to support this study are available from the corresponding author upon request.
